The article "LncRNA CTBP1-AS2 sponges miR-216a to upregulate PTEN and suppress endometrial cancer cell invasion and migration" was retracted in 2020. Reason: lack of ethics approval or compliance.

# LncRNA CTBP1-AS2 sponges miR-216a to upregulate PTEN and suppress endometrial cancer cell invasion and migration

**DOI:** 10.1186/s13048-020-00639-2

**Published:** 2020-04-15

**Authors:** Qing-an-zi Wang, Yongxiu Yang, Xiaolei Liang

**Affiliations:** Department of Obstetrics and Gynecology, Key Laboratory for Gynecologic Oncology Gansu Province, the First Hospital of Lanzhou University, Lanzhou City, Gansu Province 730000 PR China

**Keywords:** CTBP1-AS2, Endometrial carcinoma, Survival, miR-216a, PTEN

## Abstract

**Background:**

Although lncRNA CTBP1-AS2 has been functionally analyzed only in cardiomyocyte hypertrophy and diabetes, analysis of TCGA dataset revealed its downregulation in endometrial carcinoma (EC), indicating its involvement in EC.

**Results:**

In this study we found that CTBP1-AS2 was downregulated in EC and correlated with poor survival. MiR-216a might form base pairs with CTBP1-AS2 based on RNA-RNA interaction, which was confirmed by luciferase activity assay. Interestingly, upregulation of PTEN was observed after CTBP1-AS2 overexpression. Transwell assay showed that CTBP1-AS2 and PTEN overexpression led to decreased cancer cell invasion and migration and reduced enhancing effects of miR-216a on cell invasion and migration. It was known that miR-216a targeted PTEN.

**Conclusion:**

Therefore, CTBP1-AS2 may sponge miR-216a to upregulate PTEN, thereby suppressing endometrial cancer cell invasion and migration.

## Background

Endometrial carcinoma (EC) is the most commonly diagnosed gynecologic malignancies that develops from endometrium [1]. EC mostly affects menopausal females and causes a series symptoms including pelvic pain, pain with urination and vaginal bleeding [2]. Obesity is the main risk factor for EC [3]. Besides that, other factors, such as high blood pressure, excessive estrogen exposure and diabetes, are also closely correlated with the occurrence of EC [3, 4]. Based on the clinical symptoms and risk factors, early detection of EC is possible in some cases with the operation of physical examinations, such as pelvic examination, endometrial biopsy, magnetic resonance imaging and so on [5, 6]. However, these exams are not practical for all cases and early detection rate of EC is still low.

Molecular alterations are critical players in the pathogenesis of EC [7]. Functional analysis of molecular regulators in EC would facilitate the development of novel anti-EC approaches, such as targeted therapies, which aim to suppress cancer development by regulating cancer-related gene expression [8, 9]. Long non-coding RNAs (lncRNAs) are not involved in protein synthesis but can regulate gene expression at multiple levels to participate in human diseases, including cancers [10]. LncRNAs interact with cancer-related proteins and other non-coding RNAs, such as miRNAs [11]. Therefore, regulating the expression of cancer-related lncRNAs will also contribute to cancer treatment. CTBP1-AS2 has been characterized as a critical player in type 2 diabetes and cardiomyocyte hypertrophy [12, 13]. However, its involvement in cancer biology is unknown. We analyzed the expression of CTBP1-AS2 by TCGA dataset, and observed downregulation of CTBP1-AS2 in EC tissues. In addition, CTBP1-AS2 is predicted to interact with miR-216a, which can target PTEN to promote cancer development [14]. This study was therefore carried out to analyze the interactions among CTBP1-AS2, miR-216a and PTEN in EC.

## Methods

### Tissue acquisition

Paired EC tumor and non-tumor tissues were collected from 62 EC patients (47 to 68 years, 58.1 ± 4.7 years) through fine needle biopsy. All patients were enrolled at the First Hospital of Lanzhou University between January 2012 and January 2014. This study was approved by aforementioned hospital Ethics Committee. All tissue specimens were confirmed by performing histopathological exam. All the patients were excluded from other severe clinical disorders. All patients were diagnosed for the first time and no recurrent EC cases were included. All patients provided informed consent.

### Treatment and follow-up

Patients were treated with different therapeutic approaches, such as chemotherapies, radio therapies and surgeries. According to AJCC staging criteria the 62 patients included 12, 21, 18 and 11 cases at clinical stage I, II, III and IV, respectively. A 5-year follow-up was performed on all patients since the date of admission. The patients’ survival was recorded and all patients completed follow-up.

### Cells and transfections

HEC-1 (ATCC, USA) human EC cell line was used. Dulbecco’s modified Eagle’s medium (90%) was mixed with 10% FBS to prepare cell culture medium. Cells were cultivated at 37 °C in a 5% CO_2_ incubator to reach about 85% confluence.

Constructions of CTBP1-AS2 and PTEN expression vectors were performed using pcDNA3.1 vector as backbone. MiR-216a mimic and negative control (NC) miRNA were bought from Sigma-Aldrich. HEC-1 cells were transfected with CTBP1-AS2 or PTEN expression vector (10 nM) or miR-216a mimic (40 nM) using lipofectamine 2000 (Invitrogen). Cells were transfected with NC miRNA or empty pcDNA3.1 vector to be used as NC cells. Control cells(C group) were untransfected. Subsequent experiments were carried out 48 h later.

### Luciferase activity assay

Construction of CTBP1-AS2 vector was performed using pGL3 luciferase reporter vector (basic, Promega Corporation) as backbone. Lipofectamine 2000 (Invitrogen) was used to transfect HEC-1 cells with the combination of CTBP1-AS2 vector+miR-216a (miR-216a group) or the combination of CTBP1-AS2 vector+NC miRNA (NC group). Measurement of luciferase activity was performed at 48 h post-transfection using Luciferase Assay System (BPS Bioscience).

### RNA extraction

Extractions of total RNAs and miRNAs from tissue samples and HEC-1 cells were performed using RNAzol (Sigma-Aldrich) and High Pure miRNA Isolation Kit (Sigma-Aldrich), respectively. Genomic DNA was removed using gDNA eraser (Takara). NanoDrop 2000 (Thermo Scientific) was used to measure RNA concentrations and 6% urine-PAGE gel was used to check RNA integrity.

### RT-qPCR assay

BlazeTaq™ One-Step SYBR Green RT-qPCR Kit (Genecopoeia) was used to measure the expression levels of CTBP1-AS2 and PTEN mRNA. All-in-One™ miRNA qRT-PCR Reagent Kit (Genecopoeia) was used to measure the expression levels of miR-216a. GAPDH was used as the endogenous control of CTBP1-AS2 and PTEN mRNA. U6 was used as endogenous control of miR-216a. All steps were completed following manufacturer’s instructions. Three replicates were included in each experiment and ΔΔCt method was used to calculate fold changes of the levels of gene expression.

### Western blot

Total protein extractions from HEC-1 cells were performed using RIPA solution (Invitrogen) and protein samples were quantified using BCA assay (Invitrogen). Protein samples were incubated with boiling water for 15 min to achieve protein denaturation. SDS-PAGE gel (10%) was used to separate different proteins, and PVDF membranes were used to transfer proteins. PBS with non-fat milk (5% non-fat milk) was used to block membranes, followed by using GAPDH (ab9485, Abcam) and PTEN (ab31392, Abcam) primary antibodies to incubate with the membranes for 15 h at 4 °C. After that, membranes were used to incubate with HRP Goat Anti-Rabbit (IgG) secondary antibody (ab97051, Abcam) for another 2 h at room temperature. Signals were produced using ECL (Sigma-Aldrich) and were normalized using Quantity One software.

### Transwell assays

Transwell filters (8 μm; Dojindo) were used to perform Transwell invasion and migration assays using Matrigel-coated membranes and un-coated membranes, respectively. HEC-1 cells were transferred to the upper Transwell chamber (5000 cells in 0.1 ml per well), and the lower chambers contained a mixture of 20% FBS and 80% medium. Cells were cultivated at 37 °C for 12 h. After that, lower surface of membranes was stained with crystal violet (0.1%) for 20 min. Invading and migrating cells were observed under a light microscope.

### Statistical analysis

All aforementioned experiments were performed in triplicates and data were expressed as mean values. Paired t test was used to compare EC and non-tumor tissues. Luciferase activity was compared by unpaired t test. Comparisons among multiple groups were performed using ANOVA (one-way) and Tukey test. The 62 patients were grouped into high and low CTBP1-AS2 level groups (31 patients for each group). Survival curves were plotted using GraphPad Prism 6 software. Comparison of survival curves was performed using log-rank test. *P* < 0.05 was statistically significant.

## Results

### CTBP1-AS2 was downregulated in EC and correlated with poor survival

TCGA dataset was explored to analyze the expression of CTBP1-AS2. It was observed that the level of CTBP1-AS2 expression was lower in EC tissues than in non-tumor tissues (7.69 vs. 10.00). what’s more, expression levels of CTBP1-AS2 in both EC and non-tumor tissues from the total 62 patients were measured by performing RT-qPCR. Paired t test showed that expression levels of CTBP1-AS2 were significantly lower in EC tissues than in non-tumor tissues (Fig. 1a, *p* < 0.001). Survival curves were plotted for both high and low CTBP1-AS2 level groups (*n* = 31). Log-rank test analysis showed that patients in low CTBP1-AS2 level group experienced significantly lower overall survival rate (Fig. 1b).

**Fig. 1:** CTBP1-AS2 was downregulated in EC and correlated with poor survival. Expression levels of CTBP1-AS2 in both EC and non-tumor tissues from the 62 patients were measured by performing RT-qPCR. All PCR reactions were expressed as mean values and were compared by paired t test (**a**).***,*p* < 0.001. The 62 patients were grouped into high and low CTBP1-AS2 level groups (31 patients for each group). Survival curves were plotted using GraphPad Prism 6 software. Comparison of survival curves was performed using log-rank test (**b**)

### CTBP1-AS2 and miR-216a could interact with each other

The possible base pairs formed by CTBP1-AS2 and miR-216a were predicted using IntaRNA. It was observed that CTBP1-AS2 and miR-216a could form strong base pairing (Fig. 2a). Luciferase activity assay was performed by transfecting HEC-1 cells with the combination of CTBP1-AS2 vector+miR-216a (miR-216a group) or the combination of CTBP1-AS2 vector+NC miRNA (NC group). It was observed that relatively luciferase activity was significantly lower in miR-216a group than in NC group (Fig. 2b, *p* < 0.05).

**Fig. 2:** CTBP1-AS2 and miR-216a could interact with each other. The possible base pairs formed by CTBP1-AS2 and miR-216a were predicted using IntaRNA (**a**). Luciferase activity assay was performed by transfecting HEC-1 cells with the combination of CTBP1-AS2 vector+miR-216a (miR-216a group) or the combination of CTBP1-AS2 vector+NC miRNA (NC group). Mean values of 3 biological replicates were calculated and compared by unpaired t test (**b**).*,*p* < 0.05

### CTBP1-AS2 overexpression resulted in upregulation of PTEN

HEC-1 cells were transfected with CTBP1-AS2 expression vector or miR-216a mimic to analyze the interactions between CTBP1-AS2 and miR-216a. Expression levels of CTBP1-AS2 and miR-216a were significantly increased at 48 h post-transfection compared to C and NC groups (Fig. 3a, *p* < 0.05), indicating successful transfection. Comparing to C and NC groups, CTBP1-AS2 and miR-216a overexpression did not significantly affect the expression of each other (Fig. 3b). This observation suggested that CTBP1-AS2 might be an endogenous sponge of miR-216a. Therefore, qPCR and western blot were performed to analyze the effects of CTBP1-AS2 and miR-216a overexpression on the expression of PTEN at mRNA (Fig. 3c) and protein (Fig. 3d) levels, respectively. It was observed that miR-216a overexpression led to downregulated PTEN (*p* < 0.05). CTBP1-AS2 overexpression led to upregulation of PTEN (*p* < 0.05).

**Fig. 3:** CTBP1-AS2 overexpression resulted in upregulation of PTEN. HEC-1 cells were transfected with CTBP1-AS2 expression vector or miR-216a mimic to analyze the interactions between CTBP1-AS2 and miR-216a. Overexpression of CTBP1-AS2 and miR-216a was confirmed at 48 h post-transfection (**a**). The effects of CTBP1-AS2 and miR-216a overexpression on expression of each other were analyzed by qPCR (**b**). QPCR and western blot were performed to analyze the effects of CTBP1-AS2 and miR-216a overexpression on the expression of PTEN at mRNA (**c**) and protein (**d**) levels, respectively. Mean values of 3 biological replicates were calculated and compared by unpaired t test.*,*p* < 0.05

### CTBP1-AS2 interacted with miR-216a/PTEN axis to suppress EC cell invasion and migration

Comparing to C group, miR-216a overexpression caused the increased invasion (Fig. 4a) and migration (Fig. 4b) rates of HEC-1 cells (*p* < 0.05). In addition, CTBP1-AS2 and PTEN overexpression led to decreased cancer cell invasion and migration and reduced enhancing effects of miR-216a on cell invasion and migration (*p* < 0.05).

**Fig. 4:** CTBP1-AS2 interacted with miR-216a/PTEN axis to suppress EC cell invasion and migration. Transwell assays were performed to analyze the effects of CTBP1-AS2, miR-216a and PTEN overexpression on the invasion (**a**) and migration (**b**) of HEC-1 cells. Mean values of 3 biological replicates were calculated and compared by unpaired t test.*,*p* < 0.05

## Discussion

We analyzed the involvement of CTBP1-AS2 in EC. We found that CTBP1-AS2 was downregulated in EC and had predictive values for EC. In addition, CTBP1-AS2 might harbor miR-216a to upregulate PTEN, thereby inhibiting the invasion and migration of EC cells.

Previous studies have reported the involvement of CTBP1-AS2 in type 2 diabetes and cardiomyocyte hypertrophy [12, 13]. Decreased expression level of CTBP1-AS2 was closely correlated with the occurrence of type 2 diabetes and cardiomyocyte hypertrophy among Iranian population [12]., Luo et al. reported that CTBP1-AS2 could be induced by Sp1 and it could stabilize TLR4 through the interaction with FUS to participate in the disease progression [13]. Our study is the first to report the involvement of CTBP1-AS2 in cancer biology. We reported that CTBP1-AS2 was downregulated in EC and its overexpression led to inhibiting cancer cell invasion and migration. Therefore, CTBP1-AS2 was likely a tumor suppressor in EC. It was worth noting that by analyzing TCGA dataset we noticed the altered expression of CTBP1-AS2 in EC. The involvement of CTBP1-AS2 in other cancers remains to be further analyzed.

With the development of novel anti-cancer therapies, survival of early stage EC has been significantly improved [15]. However, the therapeutic effects of advanced EC remain unsatisfactory owing to the lack of effective anti-cancer therapies [16]. As an alternative approach, accurate prognosis may improve patients’ survival by guiding the selection of therapeutic approaches and care programs. Our study proved that downregulation of CTBP1-AS2 was closely correlated with the poor survival of EC patients. However, our study is limited by the small sample size. More studies with bigger sample size are needed to further test the reliability.

The function of miRNA sponge is to inhibit the function of the miRNA, but may or may not regulate the expression of the miRNA. Our data supports the idea that CTBP1-AS2 may be an endogenous sponge of miR-216a. This is based on the observation that CTBP1-AS2 and miR-216a cannot regulate the expression of each other. In addition, CTBP1-AS2 overexpression reduced the effects of miR-216a overexpression on PTEN expression, thus resulted in reducing EC cells invasion as well as migration. PTEN plays tumor suppressive roles in different types of cancers mainly by inducing cell apoptosis and suppressing cancer metastasis [14]. Therefore, PTEN may serve as the downstream effector of CTBP1-AS2/miR-216a pathway to suppress the metastasis of EC. However, other mechanisms may mediate the interactions between CTBP1-AS2 and miR-216a, future studies are still needed.

In conclusion, upregulated of CTBP1-AS2 in EC could sponge miR-216a to upregulate the expression of PTEN, thereby suppressing endometrial cancer cell migration and invasion.

## Data Availability

The analyzed data sets generated during the study are available from the corresponding author on reasonable request.

## Abbreviations

EC: Endometrial carcinoma
lncRNAs: Long non-coding RNAs
